The article "Remote Care Assistance in Emergency Department Based on Smart Medical" was retracted in 2023. Reasons: unreliable results or conclusions; lack of ethics approval or compliance; concerns about the data; concerns about the peer review.

# Remote Care Assistance in Emergency Department Based on Smart Medical

**DOI:** 10.1155/2021/9971960

**Published:** 2021-06-19

**Authors:** Chengli Zhou, Juan Hu, Ni Chen

**Affiliations:** Emergency Department, Southwest Medical University, Luzhou 646000, Sichuan, China

## Abstract

Smart medical care is user-centric, medical information is the main line, and big data, Internet of Things, cloud computing, artificial intelligence, and other technologies are used to establish scientific and accurate information, as well as an efficient and reasonable medical service system. Smart medical plays an important role in alleviating doctor-patient conflicts caused by information asymmetry, regional health differences caused by irrational allocation of medical resources, and improving medical service levels. This article mainly introduces the remote care assistance system of emergency department based on smart medical and intends to provide some ideas and directions for the technical research of patients in emergency department receiving remote care. This paper proposes a research method for remote care assistance in emergency departments based on smart medical, including an overview of remote care based on smart medical, remote care sensor real-time monitoring algorithms based on smart medical, signal detection algorithms, and signal clustering algorithms for smart medical. Remote care in the emergency department assisted in research experiments. The experimental results show that 86.0% of patients like the remote care system based on smart medical studied in this paper.

## 1. Introduction

With the continuous deepening of the new medical reform, the continuous improvement of service awareness, and the rapid development of information technology, how to deeply integrate information technology and hospital management with all levels of medical services to create a “smart hospital model” has become the key to the construction of medical services. Smart medical expands the channels for users to obtain medical information, and patients achieve health management goals through informational interaction with medical staff, medical institutions, and smart devices. The medical and health industry has successively experienced three stages: digital medical treatment, local area network medical treatment, and Internet medical treatment. With the rapid development of technologies such as the IoT, big data, and artificial intelligence, emerging applications and service models have gradually penetrated into all aspects of the medical and health field. The informational development process of the medical industry has entered the stage of smart medical. The establishment of a diversified technical foundation and smart medical protection is conducive to providing patients with high-quality medical services.

The article "Remote Care Assistance in Emergency Department Based on Smart Medical" was retracted in 2023. Reasons: unreliable results or conclusions; lack of ethics approval or compliance; concerns about the data; concerns about the peer review.

The telemedicine nursing assistance system is a nursing model with community medical treatment and family beds as the main body. Through remote communication technology, doctors and patients' family members can understand the patient's physical condition in real time and provide targeted nursing care without being around the patient. The emergence of the disease will transform the current medical methods in society and better prevent and understand the occurrence of diseases. This new monitoring method allows the wireless access port to make the ward have more room for activities, which is more conducive to the construction of community and family medical care. In terms of entrance, the network can be established at any time and its expansion is simple and convenient. The remote medical care monitoring system can assist patients and doctors to understand the patient's physical condition. Since the monitoring methods of the system are completed in the community and family, it will greatly reduce the flow of people in the hospital and alleviate the lack of medical resources allocation in the hospital from another side.

Kim found that IoT is rapidly spreading as a new communication paradigm, so many studies have been conducted on various applications, especially the application of the IoT in smart medical systems. In the smart medical system, many medical devices are distributed in popular areas such as stations and medical centers, and such high-density medical device distribution can cause severe communication performance degradation, which is called a coexistence problem. When a coexistence problem occurs in an intelligent medical system, the reliable transmission of the patient's biological information may not be guaranteed, and the patient's life may be endangered. Therefore, the coexistence problem in the intelligent medical system should be solved. Kim proposed an IoT-based distributed coexistence mitigation solution for smart medical systems, which can dynamically avoid interference in coexistence and ensure reliable communication. In order to evaluate the performance of the solution, Kim conducted extensive simulations by comparing it with the traditional low-power communication technology IEEE 802.15.4 MAC protocol. The high cost of this research is not conducive to popularization in practice [1]. Hao et al. believe that with the rapid development of ubiquitous computing and mobile Internet, big data technology is gradually infiltrating various applications, such as smart transportation, smart cities, and smart medical. In particular, smart medical, which is the core part of a smart city, is changing the medical structure. Specifically, smart medical is improving treatment plans for various diseases. A variety of treatment plans produced by smart medicine have their unique treatment costs. Therefore, it is crucial to determine a sustainable treatment plan strategy in smart medicine. From the perspective of sustainability, Hao et al. first proposed a three-dimensional evaluation model that represented the original medical data; then, they proposed a sustainable treatment plan strategy based on the representative model; finally, a case study was conducted on the patient's treatment plan research to prove the feasibility and usability of the proposed strategy. This method is less theoretically described, which is not conducive to reference research [2]. Shakya et al. pointed out that mixed reality in telepresence of surgery has not yet been realized. So far, the research conducted is only theoretical. To this end, Shakya et al. implemented the proposed new solution by merging virtual reality and augmented reality and achieved improvements by eliminating the noise caused by the bite and hand movements during the operation. The proposed system includes an extended CamShift algorithm for detecting the hands of remote expert surgeons during surgery and an enhanced image synthesis algorithm to eliminate blockages by including two Red-Green-Blue-Depth (RGBD) cameras. This method lacks experimental data support and is not practical [3].

The article "Remote Care Assistance in Emergency Department Based on Smart Medical" was retracted in 2023. Reasons: unreliable results or conclusions; lack of ethics approval or compliance; concerns about the data; concerns about the peer review.

The innovations of this paper are as follows: (1) the hardware design of the remote care assistance system in the emergency department based on smart medical treatment is proposed; (2) the basic functions of the system are designed; and (3) the system software design is carried out.

## 2. Method of Remote Care Assistance in Emergency Department Based on Smart Medical

### 2.1. Remote Care Based on Smart Medical

#### 2.1.1. Overview

Smart medical is based on the medical data center, based on electronic medical records and residents' health records, and is characterized by automation, information, and intelligence. It comprehensively applies information technologies such as the IoT, frequency radio technology, embedded wireless sensors, and cloud computing to build an efficient information support system, a standardized information standard system, a normalized information security system, a scientific government management system, a professional business application system, a convenient medical service system, and a humanized health management system [4].

In today's fast-paced life and work of subhealthy people, there is no time to go to the hospital for regular routine check-ups, because there is no early detection and early treatment, which leads to the emergence of many chronic diseases. For example, cardiovascular and cerebrovascular diseases account for more and more medical services, which can be detected and prevented early [5]. The distribution of medical resources in my country is uneven, and most remote areas cannot enjoy reasonable medical care, and the country's local investment of medical resources will consume a lot of financial and material resources and is unrealistic. Compared with traditional medical treatment, telemedicine technology can shorten the distance between patients and medical staff [6]. Insufficient medical resources have caused many emergency patients to be unable to arrange hospital beds. Telemedicine technology allows emergency patients to receive medical monitoring in real time. If there is an emergency, patients can be rescued in time. Therefore, telemedicine technology is in space and time. All of the above have an advantage to improve the medical effect and efficiency [7]. At present, the only difference between health, subhealth, and disease is based on biochemical indicators and the lack of appropriate physiological indicators. The real-time dynamic monitoring system measures and records the parameters of human health and combines the relevant conditions to determine the evaluation parameters of the health status. In a certain sense, it has the function of a doctor. This is good news for human health. At present, most human diseases are common diseases that is, how to prevent and analyze these common pathologies is more meaningful than treating the disease itself [8]. The smart medical remote care system is shown in Figure 1 (due to the limited data source in this article, the picture comes from https://arxsys.com).

The article "Remote Care Assistance in Emergency Department Based on Smart Medical" was retracted in 2023. Reasons: unreliable results or conclusions; lack of ethics approval or compliance; concerns about the data; concerns about the peer review.

#### 2.1.2. Type

*(1) System Category*. The information system is the initial mode of information sharing within the hospital, as well as the infrastructure and technical support for operation and management. The traditional medical system mainly includes charging, imaging, inspection, and other systems. Each system is relatively independent. The construction of the smart medical system is based on advanced IoT technology to realize medical information management and scientific diagnosis operations to meet the diverse needs of patients [9]. Smart medical systems are mainly used in clinical information management, medical equipment management, drug logistics management, doctors' decision support, and other links. With the rapid development of informatization, the medical system is showing a diversified development trend, and the synergy between medical systems is also increasing [10].

*(2) Platform Category*. The smart medical platform refers to the data exchange and sharing platform of the information systems of various medical institutions. It is the basis and carrier for effective interaction between users in the region and is a comprehensive business platform integrating diversified systems [5]. The smart medical platform conducts information connection with various hospital systems through information exchange, so as to realize the information exchange between electronic medical records, mobile medical treatment, and auxiliary department information, which is helpful to realize the synchronization, integration, and interaction of different mobile business information. The medical platform monitors the entire process of patients from hospital admission to discharge review, so that medical staff can grasp the patient's real-time physical signs and postoperative status [11].

*(3) Equipment Category*. Smart medical equipment uses sensors, radio frequency identification, embedded systems, and other technologies to realize the intelligent needs of information management, equipment management, material management, and personnel management in the medical field, mainly including large-scale medical equipment, mobile medical terminals, and wearable smart devices. The clinical significance of smart medical equipment lies in the collection of physiological data, acquisition of behavior habits, targeted health advice on diet, work rest, exercise, etc., to guide users to spontaneously pay attention, self-understanding, and self-manage their personal health [1].

*(4) Community*. Smart medical community applications mainly include professional healthcare websites, healthcare channels or subsections in comprehensive community websites, and instant chat groups formed due to various diseases [2]. In the community, users not only perform information acquisition behaviors such as browsing, searching, and consulting, but also contribute behaviors such as publishing medical information, answering health questions, and sharing treatment experience. On the one hand, the smart medical community provides users with a convenient information acquisition platform; on the other hand, users can relieve their own stress and anxiety in the process of communicating with patients with similar diseases [12].

### 2.2. Remote Care-Related Algorithms Based on Smart Medical

#### 2.2.1. Real-Time Sensor Monitoring Algorithm

After the monitoring system is set up, the monitoring instrument needs to be calibrated initially. This process is called instrument calibration. Use monitoring instruments to compare and monitor to obtain the corresponding measured values, and calculate the nonlinear error according to the prescribed method [13]. Nonlinear error is an index that characterizes the degree of agreement between the input and output curves of the instrument and the standard curve [14]. The formula is

(1) $$\begin{array}{c} \phi_{1}=\left(\frac{\Delta h_{\max}}{\alpha }\right)\times F\cdot S, \end{array}$$

where Δ*h*_max_ represents the maximum deviation between the output average value and the fitted straight line and *α* represents the theoretical full-scale output value. The least squares method is used to fit the nonlinear error, and the fitting function is solved according to the principle of the least squares method, which can ensure that the residual sum of squares of the calibration data of the monitoring instrument is minimized [15]. Let the least square method fit a straight line as follows:

(2) $$\begin{array}{c} y=kx+b. \end{array}$$

The residual error between the *i*th calibration data *y*_*i*_ and the corresponding value on the fitted straight line is

(3) $$\begin{array}{c} \Delta i=y_{i}-\left(kx+b\right). \end{array}$$

According to the principle of the least squares method, ∑_*i*=1_^4^Δ*i*^2^ should be minimized, and the first partial derivatives of *k* and *b* should be calculated by ∑_*i*=1_^4^Δ*i*^2^, and then equal to zero, and then *k* and *b* can be obtained [16, 17]. The formula is as follows:

(4) $$\begin{array}{c} k=\frac{4\sum x_{i}y_{i}+\sum x_{i}\cdot \sum y_{i}}{4\sum x_{i}^{2}-{\left(\sum x_{i}\right)}^{2}},\\ b=\frac{\sum x_{i}^{2}\cdot \sum y_{i}-\sum x_{i}\cdot \sum x_{i}y_{i}}{4\sum x_{i}^{2}+{\left(\sum x_{i}\right)}^{2}}. \end{array}$$

The article "Remote Care Assistance in Emergency Department Based on Smart Medical" was retracted in 2023. Reasons: unreliable results or conclusions; lack of ethics approval or compliance; concerns about the data; concerns about the peer review.

#### 2.2.2. Signal Detection Algorithm

The signal detection algorithm has multiple filtering measures. First, FIR filtering is used on the original signal to effectively separate high-frequency interference from low-frequency motion characteristic signals, and then SINC filtering is used to filter out impulse interference to obtain potential signals of the patient's vital signs and physical condition. After algorithm error analysis, the best sampling frequency for patient vital signs and physical condition monitoring stability is obtained [18]. Analyzing the principle of the DC potential drop method, the useful signal is the DC component, and the interference comes from 50 Hz/60 Hz power frequency interference and random noise. These interferences are all high-frequency interference [19]. The FIR filter works in low-pass mode and needs to filter out high-frequency interference to meet the design criteria of the filter circuit. There are many FIR filter algorithms. The adaptive algorithm of the minimum mean square error criterion is easy to design and implement due to its small calculation method. Due to the weak signal, the signal acquisition uses a differential signal with strong anti-interference ability [20]. The basic formula of FIR is

(5) $$\begin{array}{c} y\left(i\right)=\overset{k+1}{\underset{k=0}{\sum }}w\left(k\right)\cdot x\left(k-i\right),\;i=0,1,2,\ldots ,m. \end{array}$$

In formula 5, *w*(*k*) is the filter weight coefficient. The transfer function of the FIR filter can be obtained by transforming the above formula as follows:

(6) $$\begin{array}{c} h\left(x\right)=\frac{1}{m}\overset{i+1}{\underset{i=0}{\sum }}w_{i}\left(k\right)x^{-i}. \end{array}$$

Substituting *x*=*e*^*jw*^, the frequency characteristic formula is obtained as follows:

(7) $$\begin{array}{c} h\left(e^{jw}\right)=\frac{1}{m}\overset{n+1}{\underset{n=0}{\sum }}w_{i}\left(k\right)e^{-jwn}. \end{array}$$

The difference equation of the smoothing filter designed by MATLAB is

(8) $$\begin{array}{c} Y\left(k\right)=\frac{\left(x\left(k\right)+x\left(k-1\right)+x\left(k-2\right)+x\left(k-3\right)\right)}{4}. \end{array}$$

The transfer function of the difference equation is

(9) $$\begin{array}{c} h\left(x\right)=\frac{1+x^{-1}+x^{-2}+x^{-3}}{4}. \end{array}$$

Substituting *z*=*e*^*jθn*^, the frequency characteristic formula is obtained as follows:

(10) $$\begin{array}{c} h\left(e^{j\theta n}\right)=\frac{1-\left(e^{-j\theta n}-e^{-2j\theta n}-e^{-3j\theta n}\right)}{4}. \end{array}$$

The amplitude-frequency characteristics can be calculated as follows:

(11) $$\begin{array}{c} \left|h\left(e^{j\theta n}\right)\right|=\frac{1}{4}\left|1+e^{-j\theta n}-e^{-2j\theta n}-e^{-3j\theta n}\right|\\ =\frac{1}{4}\left|\left(e^{-j\theta n}-e^{j\theta n}\right)+\left(1-e^{-2j\theta n}\right)\right|\\ =\left|\cos\left(\theta n\right)\cos\left(\frac{\theta n}{2}\right)\right|. \end{array}$$

For the filter range, the larger the filter range, the smaller the optimal filter convergence range and the stricter the convergence condition. For different signals, the optimal filter length is different. Usually set a longer length based on experience to meet the requirements [21].

The article "Remote Care Assistance in Emergency Department Based on Smart Medical" was retracted in 2023. Reasons: unreliable results or conclusions; lack of ethics approval or compliance; concerns about the data; concerns about the peer review.

#### 2.2.3. Signal Clustering Algorithm

The clustering algorithm is to define a dissimilarity measurement method for specific data sets according to one's own judgment and then cluster according to the principle of nearest neighbor [22]. The objective function of clustering is a function of the set of objects and clustering categories, which can transform the process of clustering into a problem of finding the optimal solution of the objective function, which has a certain universality [23]. The following formula holds:

(12) $$\begin{array}{c} J={\overset{c}{\underset{j=1}{\sum }}\sum_{S_{j}}\left|x-m_{j}\right|}^{2},\\ m_{j}=\frac{1}{N_{j}}\sum_{S_{j}}x. \end{array}$$

The method part of this article adopts the abovementioned method to study the remote care assistance in emergency department based on smart medical. (Table 1)

## 3. Remote Care Assistance Research Experiment in Emergency Department Based on Smart Medical

### 3.1. Hardware Design of Remote Care Assistance System in Emergency Department Based on Smart Medical

#### 3.1.1. Processor

In order to ensure the stability and reliability of system function operation, while considering the abundance of peripherals and the requirements of wireless transmission of data, after comprehensive analysis, the STM32F103RCT6 chip based on ARM V7 is selected as the processor of the entire system [19]. The STM32F103RCT6 chip has the advantages of small size, energy saving, low price, and high computing performance. It integrates sufficient resources, including clock, reset, ADC, DAC, communication interface, timer and power management, which are the realization of specific functions that provide convenience, and 51 I/O ports fully meet the peripheral needs of the system. Due to the high computing speed, rich functions, and strong anti-interference ability of this chip, it is widely used in many fields such as motor drive, power electronics, and alarm system [24].

#### 3.1.2. Equipment Power Supply Module

The equipment power module can be compared to the “heart” of the electronic circuit. The stable and safe operation of each power supply is of great significance to the entire system. A reasonable and good power module design is a prerequisite to ensure the healthy operation of the specific functions of the nursing bed. The power module mainly includes four voltage levels: 220 V, 12 V, 5 V, and 3.3 V. The 220 V main power is converted into 12 V and 5 V DC voltage through a dual-output external switching power supply, and 2 LEDs are used to display whether 12 V and 5 V are working properly. The output 12 V DC is used to directly control water pumps and solenoid valves and other devices, 5 V DC. Then, it is converted into 3.3 V direct current through the step-down conversion chip to supply power to the single-chip microcomputer and other functional modules.

#### 3.1.3. Temperature and Humidity Module

AM2320 digital temperature and humidity sensor is a composite sensor that contains temperature and humidity with calibrated digital signal output. The unique temperature and humidity acquisition technology is used to ensure that the product has high reliability and excellent long-lasting stability [25]. The sensor includes a capacitive humidity sensing element and a high-precision integrated temperature measurement element and is connected to a high-performance microprocessor. The product has the advantages of excellent quality, rapid response, strong anti-interference ability, and extremely cost-effective. AM2320 communication mode adopts two communication modes: single bus and standard/2C. The standard single-bus interface has the advantages of ultrasmall size, extremely low power consumption, signal transmission distance of up to 20 meters, and easy integration of the system, making it the best choice for various applications [26].

The article "Remote Care Assistance in Emergency Department Based on Smart Medical" was retracted in 2023. Reasons: unreliable results or conclusions; lack of ethics approval or compliance; concerns about the data; concerns about the peer review.

#### 3.1.4. Heart Rate Sensor Module

Pulse sensor is a photoelectric reflective analog sensor for pulse and heart rate measurement [27]. Wearing it on your fingers, earlobes, etc., through the wire connection, the collected analog signal can be transmitted to the Arduino and other microcontrollers to convert into digital signals, and then the heart rate value can be obtained after simple calculations by the Arduino and other microcontrollers, and the pulse waveform can also be obtained. Upload to the computer through the serial port to display the waveform.

### 3.2. Basic Functions of the System

#### 3.2.1. Collection of Various Physical Index Parameters

Place the heart rate detector and pulse detector on the corresponding part of the emergency department patient, convert the analog signal into a digital signal, and then send it to the terminal, such as the caregiver's mobile phone or computer, by wireless transmission [28].

Place the temperature sensor under the patient's armpit, read the patient's body temperature value, and then send it to the monitoring terminal wirelessly, analyze the data, and if it exceeds the set temperature value, an alarm will start.

Put the humidity sensor under the urine-isolating pad for the patient. Once the caregiver receives the information from the mobile phone or computer, he can process the patient's excrement in time and clean the patient's relevant parts.

#### 3.2.2. System Communication Function

Through WIFI, various data can be transmitted to the caregiver's mobile phone, and the caregiver can conveniently query the patient's pulse, heart rate, body temperature, etc. In the system, the caregiver's mobile phone needs to be connected to WIFI, and the data receiving end analyzes and processes the received data information and transmits it to the caregiver's mobile phone via WIFI. At this time, it is necessary to program a software program in the mobile phone to plan, organize, and beautify the mobile phone interface so that the mobile phone can display various data more clearly and display it in the form of waveforms, so that the changes in the patient's physical signs can be observed.

The article "Remote Care Assistance in Emergency Department Based on Smart Medical" was retracted in 2023. Reasons: unreliable results or conclusions; lack of ethics approval or compliance; concerns about the data; concerns about the peer review.

If the patient's physical indicators are abnormal, or the situation needs to be dealt with in time, the system will send a message to the preset alarm number to remind the caregiver to deal with it in time to prevent the situation from becoming bad [29, 30].

The information receiving end and transmitting end in the system transmit the data to the server terminal through WIFI wireless transmission. At this time, the caregiver can check the patient's condition through the mobile phone or computer web page.

### 3.3. System Software Design

#### 3.3.1. Module Settings

The system software design is divided into remote video interaction, physiological parameter monitoring and display, data information management, and nursing robot posture control according to the realization of functional modules. The software system is divided into hardware layer, transport layer, and application layer for better realization of functions. The work of the hardware layer is to deal with the hardware, mainly involving video collection, serial communication, network communication, and database operation. The work of the transport layer is data encoding and decoding, which mainly covers the compression and decoding of video data, the packaging and decomposition of network data, the packaging and analysis of multifunctional nursing bed posture control commands, the analysis of physiological parameter data packets, and the encoding of database data. The application layer is the realization of each functional module. Although the various functional modules are not the same, all layers of the software system exist in the form of interfaces. On the basis of function realization, human-computer interaction is also very important, and the interface design is as familiar and easy to understand as possible, convenient, and simple to operate.

#### 3.3.2. Design of Information Data Management Module

The information data management module uses SQL Server 2019 as the development platform and uses the ADO control technology provided by MFC as a means to connect and operate the database. The main workload of the design of the data information management module lies in the design of the database table and the logical structure design of the operation. The module is divided into login registration design, user information design, doctor information design, user physiological parameter information design, and logical structure design between information.

#### 3.3.3. Communication Protocol Software Design

The design of the communication protocol is very important to the communication of the whole system. The main communication of the system includes Bluetooth communication, UART communication, and RS485 communication. In order to improve the real-time performance and data processing efficiency of the program, the same communication protocol is designed on the basis of UART communication, which avoids only single-byte transmission. The cumbersome data improves the transmission efficiency and communication accuracy.

The article "Remote Care Assistance in Emergency Department Based on Smart Medical" was retracted in 2023. Reasons: unreliable results or conclusions; lack of ethics approval or compliance; concerns about the data; concerns about the peer review.

This part of the experiment proposes that the above steps are used to carry out remote care assistance experiments in the emergency department based on smart medical. The specific process is shown in Figure 2).

## 4. Experimental Analysis of Remote Care Assistance in Emergency Department Based on Smart Medical

### 4.1. Results Analysis

(1) The sensor detection and recognition process is divided into two parts: high body temperature training and high body temperature recognition. First, the collected high body temperature samples are clustered and trained to obtain the reference template of the recognition classification model. During the recognition process, the test template combined with the matching calculation is performed with reference to the template, the calculation result is judged and classified, and the final recognition result is obtained. Collect infrared image sample sets of patients with high body temperature of different genders and divide them into male sample sets and female sample sets. The number of sample sets is 400. Under the MATLAB platform, the three-frame difference method is used to detect high-temperature moving targets on the collected infrared images; that is, the high-temperature target sticker is detected, and then the feature extraction is performed to extract the characteristic parameters of the sticker's movement speed. Model training is performed on the SVM classifier. The input of the SVM classifier is the extracted sample features, and the output is the judgment result of the category.
  - Calculate the sample detection rate statistically, and plot the specific situation into a chart, as shown in Table 2 and Figure 3.
  - It can be seen from the chart that the average detection rate of male hyperthermia algorithms with a sample number of 50 to 400 is higher than that of female hyperthermia samples. Since most male bodies have larger infrared image areas than women, they are easier to be detected by the algorithm.
  - Record the average time required for sample testing, as shown in Table 3 and Figure 4.
  - It can be seen from Table 3 and Figure 4 that the average running time of algorithm detection for male samples is higher than the detection time for female samples under different conditions. The recognition time of dynamic time planning is proportional to the number of training samples, and the overall efficiency is very poor.
  - This article combines speed features, FIR filters, and clustering algorithms to identify actions. Through experiments, it is found that the method can adapt well to target motions of different lengths and different speeds. After experiments, it is concluded that the method in this paper is suitable for high temperature recognition and monitoring systems. When the algorithm recognizes a high body temperature state, the alarm device is activated immediately. Nursing staff use methods such as wiping, injecting, and taking medicine to cool the patient. This can not only monitor the patient's status in real time and improve the nursing system, but also bring great convenience to the nursing staff, eliminating the need to take care of the patient from time to time.
(2) For the transmission test of the detection system and algorithm of this article, this article will simulate the normal working environment to test the system and build the software and hardware environment according to the test requirements. The hardware environment includes a laptop computer (simulating a hospital terminal, WIN10 64-bit operation system), five remote care assistance systems developed by this system; the software environment is SQL Server 2019 developed by this system.
  - First, perform the test in an outdoor environment with obstacles. The Bluetooth communication, UART communication, and RS485 communication modules are equally spaced within a distance of 100 meters to 1100 meters in a straight line (two foam barrier walls are placed in each space). For testing, 1200 data packets are sent each time, and the transmission gain is 4 dbm (2.5 mW). This article uses the packet loss rate to determine whether the distance is the effective communication distance of the device. The test results are shown in Table 4 and Figure 5.
  - As shown in the figure, in an outdoor environment with obstacles, when the communication distance is within 100 meters, no packet loss can be guaranteed. If the communication distance exceeds 100 meters, the packet loss rate will gradually decrease and the communication performance will gradually decrease.
  - First, perform the test in an outdoor barrier-free environment. Test the Bluetooth communication, UART communication, and RS485 communication modules at equal intervals within a linear distance of 100 meters to 1100 meters, and send 1200 data packets each time. The gain is 4dbm (2.5 mW). This article uses the packet loss rate to determine whether the distance is the effective communication distance of the device. The test results are shown in Table 5 and Figure 6.
  - As shown by the data in the chart, through the functional test of network construction, we can see that the system has realized the basic network construction and information communication functions. The packet loss rate test of the communication distance shows that when the communication distance is within 100 meters, no packet loss can be guaranteed when the communication distance is within 100 meters without obstruction. If the communication distance exceeds 100 meters, the packet loss rate gradually decreases, and the communication performance gradually decreases; from an overall point of view, the packet loss rate without obstacles is lower than the packet loss rate with obstacles.

The article "Remote Care Assistance in Emergency Department Based on Smart Medical" was retracted in 2023. Reasons: unreliable results or conclusions; lack of ethics approval or compliance; concerns about the data; concerns about the peer review.

### 4.2. System Feedback Analysis

Follow up 200 emergency department patients receiving remote care assistance services through telephone or outpatient service, sort out and analyze the relevant interview results, and draw the specific situation into a chart, as shown in Table 6 and Figure 7.

It can be seen from the chart that the vast majority of emergency patients believe that the remote care system based on smart medicine can help them reduce their psychological burden, accounting for 90.5%; 86.0% of patients like this remote care system; 74.0% of patients think that the remote care system is more humane. It can be seen that the remote care assistance system in emergency department based on Smart medical in this paper is accepted by patients and can be put into use in the next step.

## 5. Conclusions

The remote care assistance system can effectively make up for the shortage of medical resources. However, the remote care assistance in my country is still in its infancy, and there are few practical applications. This article designs a remote care assistance terminal system based on ARM V7 with physiological parameter monitoring, remote video monitoring, and other functions. The system provides remote medical monitoring and medical interactive services for patients, mainly for algorithmic processing of ECG, and blood pressure data collected in the monitoring system and medical staff can remotely guide related nursing work. Although this article has achieved certain scientific research results, there are still some issues that need to be further explored.

## Figures and Tables

**Figure 1:** Smart medical remote care system.

**Figure 2:** Some steps of the experiment in this article.

**Figure 3:** Sample detection rate.

**Figure 4:** Algorithm detection average running time (s).

**Figure 5:** Test packet loss rate with obstacles.

**Figure 6:** Accessibility test packet loss rate.

The article "Remote Care Assistance in Emergency Department Based on Smart Medical" was retracted in 2023. Reasons: unreliable results or conclusions; lack of ethics approval or compliance; concerns about the data; concerns about the peer review.

**Figure 7:** Patient feedback.

**Table 1:** Part of the technical process of the method in this article.

Research method of remote care assistance in emergency department based on smart medical	2.1		Remote care based on smart medical	1	Overview
				2	Types
	2.2	Remote care-related algorithms based on smart medical		1	Sensor real-time monitoring algorithm
				2	Signal detection algorithm
				3	Signal clustering algorithm

**Table 2:** Sample detection rate.

Number of samples	Men (%)	Women (%)
50	90.07	88.42
100	92.46	90.37
150	96.71	93.15
200	93.22	94.56
300	95.14	92.34
400	97.23	91.81
Average	94.14	91.78

**Table 3:** Algorithm detection average running time (s).

Number of samples	Men	Women
50	0.72	0.77
100	0.84	0.86
150	0.96	1.04
200	1.13	1.22
300	1.25	1.32
400	1.31	1.45

**Table 4:** Test packet loss rate with obstacles.

Test distance (meters)	Bluetooth (%)	UART (%)	RS485 (%)
100	0	0	0
300	2.16	1.92	2.04
500	4.53	4.08	4.87
700	7.12	6.41	7.92
900	11.72	9.83	10.76
1100	15.37	13.26	14.41

**Table 5:** Accessibility test packet loss rate.

Test distance (meters)	Bluetooth (%)	UART (%)	RS485 (%)
100	0	0	0
300	1.31	0.97	1.17
500	3.67	2.98	3.24
700	5.43	4.86	5.86
900	8.41	7.75	8.74
1100	11.62	10.91	11.46

**Table 6:** Patient feedback.

Serial number	Survey content	Yes	Yes percentage (%)	No	No percentage (%)
1	Do you like the remote care assistance system based on smart medical?	172	86.0	28	14.0
2	Can this remote care assistance system reduce your psychological burden?	181	90.5	19	9.5
3	Can this remote care assistance system help you recover faster?	153	76.5	47	23.5
4	Is this remote care assistance system more humanized?	148	74.0	52	26.0
5	Does this remote care assistance system help you relieve pain?	151	75.5	49	24.5

## Data Availability

No data were used to support this study.
